# *Sedum sarmentosum* Bunge Attenuates Drug-Induced Liver Injury via Nrf2 Signaling Pathway: An Experimental Verification Based on Network Pharmacology Prediction

**DOI:** 10.1155/2021/1142638

**Published:** 2021-11-02

**Authors:** Zhitao Jiang, Yi Han, Yuechan Zhang, Jie Li, Chundi Liu

**Affiliations:** Department of Pharmacy, Zhangjiagang Hospital of Traditional Chinese Medicine, Affiliated Hospital of Nanjing University of Chinese Medicine, Zhangjiagang, Suzhou, Jiangsu 215600, China

## Abstract

**Purpose:**

Using network pharmacology and in vivo experiments, we investigated the antidrug-induced liver injury components and functional processes of *Sedum sarmentosum* Bunge (SSBE).

**Methods:**

The effective components, primary active ingredients, and possible target in the therapy of DILI were predicted using network pharmacology and bioinformatics. APAP was inducing the DILI model. In vivo testing of the pharmacodynamic foundation of SSBE in the treatment of DILI was performed.

**Results:**

The TCMSP database evaluated five main active components and 299 related targets. In addition, 707 differential genes for DILI were obtained from the DisGeNET database, DigSee database, and OMIM database. 61 related targets were mapped to predict the targets of SSBE acting on DILI. The protein-protein interaction (PPI) core network contained 59 proteins, including IL-*β*, MARK14, SSP1, and MMP9. These genes are closely related to the Nrf2/ARE signaling pathway, and they may play a key role in the hepatoprotective effect of SSBE. Verification experiment results showed that, in the DILI mouse model, SSBE promoted inflammation diminution and regulation of Nrf2-ARE cascade. SSBE protected normal hepatocyte growth and inhibited apoptosis of normal liver cells induced by APAP. SSBE inhibited the expression of Nrf2 and ARE proteins in the liver tissue of the DILI mouse model in vivo.

**Conclusion:**

By modulating the Nrf2 signaling pathway, the active components in SSBE may protect against drug-induced liver damage.

## 1. Introduction

Injury to the liver caused by drugs (drug-induced liver injury (DILI)) refers to abnormalities in liver function tests related to the intake of medicinal compounds, medications, aerobatics, and herbs and is attributed to a significant percentage of patient morbidity and mortality, with an annual incidence rate between 1 and 20 per 100,000 people [1]. DILI can cause serious consequences, including hepatitis, liver fibrosis, liver failure, and even death. Around the world, drug-induced liver damage (DILI) has been a major health problem [2]. Although currently used liver parameters are sensitive, DILI still lacks simple, objective, and specific diagnostic indicators and specific treatments. The medicines for DILI that are both safe and efficacious are desperately required.

Traditional Chinese medicine (TCM) offers unique benefits for treating DILI and has been shown to have hepatoprotective effects. As a traditional medicinal plant, *Sedum sarmentosum* Bunge (SSBE) has been recorded by Chinese Pharmacopoeia (2010), and various preparations have been developed from it [3]. It is widely used in clinical application to treat many kinds of liver diseases, such as dampness-heat of liver and gallbladder and acute and chronic hepatitis. SSBE mainly contains flavonoids, mainly *Sedum sarmentosum* total flavonoids (SSTF), and other compounds, which have various biological functions such as liver protection, antitumor, anti-inflammatory, antioxidation, antikidney fibrosis, and strengthening muscle strength [4, 5].

It has been previously verified that SSBE has a protective effect on drug-induced liver injury, but few research studies have been done on the primary active ingredients and possible molecular mechanisms of action. The pathogenesis and pathological factors of drug-induced liver injury are relatively complex, with complex components and numerous targets, so how to interpret the mechanism of drug-induced liver injury more comprehensively is an urgent problem to be solved. However, single component-single target-single disease is not suitable for the study of Chinese herbal compound.

Using a variety of databases, pathway analysis, and network analysis, network pharmacology, as a new era in contemporary traditional Chinese medicine (TCM) pharmacological investigations, can be used to envisage the targets of action with TCM, discover the active components of TCM, and explore the mechanism of TCM as disease treatments [6]. Network pharmacology is based on a multidrug target network, gene network of disease in human, and PPI network, namely, drug-disease-gene multilevel network [7, 8]. Through network pharmacology, more intuitively we understand the interaction between SSBE and DILI, and we can understand and explore the possible anti-DILI mechanism of SSBE at the molecular level. Therefore, based on network pharmacology notion, this investigation intends to show the main targets of *Sedum sarmentosum* Bunge against drug-induced liver injury, so as to explore theoretical origin towards subsequent basic research on pharmacodynamic substances and their mechanism exploration. In the current investigation, network pharmacology was used to screen SSBE constituents that were effective in the treatment of DILI, and molecular biology tools were used to evaluate the potential molecular mechanism in a mouse model to provide a foundation for prospective clinical studies on the effectiveness of SSBE in the treatment of DILI.

## 2. Materials and Methods

### 2.1. SSBE Bioactive Compounds Screening

Traditional Chinese Medicine Systems Pharmacology Database (TCMSP) (http://lsp.nwu.edu.cn/tcmsp.php,Version:2.3) that offers various databases on plant components and their chemical structures [9] was used to obtain information on SSBE compounds. TCMSP also offers characteristics relating to ADME (absorption, distribution, metabolism, and excretion) of herbal constituents, such as oral bioavailability (OB), drug-likeness (DL), and half-life [10]. After data from TCMSP was gathered, OB and DL were utilised to screen bioactive components of SSBE. The rate and amount of medication absorption to the circulatory system are measured by OB, a key pharmacokinetic parameter of orally given drugs [11]. DL is a qualitative principle that may be used to assist in enhancing pharmacokinetics and pharmacological characteristics in drug development [12]. It can be used to forecast the likelihood of a chemical molecule becoming a medication. Only compounds with OB ≥30% and DL ≥0.18 were chosen for further investigation. The time it takes for the concentration of medicines in blood/the number of drugs in the body to drop to half is referred to as the half-life. It represents the rate at which medicines are eliminated from the body. The optimum condition in this research was HL ≥4 h. ADME screening was used to exclude certain chemicals for this reason. Finally, 5 active ingredients were eliminated.

### 2.2. Identifying SSBE Targets

To determine the link between each chemical component and its possible targets, we searched through the TCMSP database and Cytoscape 3.7.1 software (https://cytoscape.org/). The following two features of the database are used to obtain drug-target interactions: (1) drug targets from the HIT database that have been experimentally verified and (2) SysDT models that were mostly utilised for the prediction of drug combinations without experimental data support. Obtaining a target necessitates a more succinct statement of the connection between the active component and the target, as it involves numerous species targets. As a result, we utilised the UniProt database (http://www.uniprot.org/) to find the gene names of all targets, using humans as the chosen species.

### 2.3. Probing DILI Targets

The DILI targets were obtained from three different sources: (1) the DisGeNET database (http://www.disgenet.org/); (2) the DigSee database (http://210.107.182.61/geneSearch/); and (3) the Online Mendelian Inheritance in Man (OMIM) (http://omim.org/). Our investigation searched these human illness target databases for targets associated with DILI using the keywords “drug-induced liver damage” and the species “homo species.” The targets linked to DILI were found by searching for the term “drug-induced liver damage.” The website http://www.uniprot.org/was used to bring the targets together.

### 2.4. Network Establishment

Common targets linked to DILI and potential targets of bioactive substances were chosen as SSBE's targets against DILI in order to study the possible mechanisms of SSBE on DILI. Wayne at the website http://bioinforgp.cnb.csic.es/tools/venny/index.html set the intersection between medication active component of compound targets and illness targets. UniProt (https://www.uniprot.org/) moved all of the targets to “ENTRY” before the network was established. Cytoscape 3.7.1, an open-source software project, was used to create the networks. It integrates biomolecular interaction networks with high-throughput expression data and other molecular states into a coherent conceptual framework.

### 2.5. Pathway Analyses and Collection of PPI Data

The SSBE pathways associated with DILI were investigated using the Database for Annotation, Visualization, and Integrated Discovery (DAVID, https://david.ncifcrf.gov/home.jsp, Vision 6.8) and KEGG (https://www.kegg.jp/, Release 91.0). The results of GO and KEGG pathway enrichment were considered to have statistically significant and necessary functional mechanisms of DILI, when *P* < 0.05. Search Tool for the Retrieval of Interacting Genes (STRING, https://string-db.org/) was used to collect possible protein-protein interactions (PPI) by uploading 61 common targets that related to DILI and putative targets of active compounds. Species were limited to “*Homo sapiens*” with a confidence score >0.4.

### 2.6. Animals and Drugs

A total of 50 male ICR mice (15–20 g) were randomly assigned to 5 groups: PBS control group, APAP model group, and total flavonoids drug preconditioning group (low dose 50 mg/kg, medium dose 100 mg/kg, and high dose 200 mg/kg). The rats were given intraperitoneal injection of APAP 1 h after the last administration of SCF extract. At the end of the experiment, all animals were sacrificed for subsequent analysis.

### 2.7. Pathological Score and Liver Segment

The tissue samples of mice liver were preserved in 4% neutral formaldehyde, dried, and paraffin-embedded. The fossils were cut into four-meter thick slabs and dyed with HE. The pathological alterations in the pancreas following HE staining were examined under a light microscope and scored using the METAVIR pathological score as a guide.

### 2.8. ELISA

The concentrations of amylase, ALT, and AST in animal serum or cell culture medium were detected using an ELISA kit according to the manufacturer's instructions. GST/SOD activities and GSH/MDA contents were detected by the biochemical method.

### 2.9. Western Blot and QT-PCR

The expression of Nrf2/ARE protein in each group was determined by Western blotting. The changes of Nrf2/ARE mRNA levels in normal liver cells treated by APAP were determined by QT-PCR. To separate the proteins, a suitable lysis solution was employed, and the protein content was determined using a BCA assay kit. The protein sample was separated on a 10% SDS-polyacrylamide gel (SDS-PAGE), and the proteins were then transferred to a PVDF membrane. The membrane was blocked with 10% BSA for 120 minutes before being incubated at 4°C overnight with the target antibodies and the GAPDH antibody as the reference protein. The membrane was rinsed three times in TBST for 10 minutes before being incubated for two hours at room temperature with sheep anti-rabbit IgG secondary antibody. The membrane was rinsed three times with TBST for ten minutes before being imaged with ECL photoluminescence solution. The test data were analysed using ImageJ software. Total RNA was isolated from single E10.5 embryos using the TRIZOL reagent (Life Technologies) and the guanidine isothiocyanate technique for quantitative PCR (QT-PCR).

### 2.10. CCK8 Assay and Flow Cytometer Detection

The CCK8 test was used to determine cell viability. Cell Counting Kit 8 (CCK8, Dojindo, Japan) was used for the CCK8 test according to the manufacturer's instructions. In all groups, flow cytometry was utilised to identify LO2 apoptosis in normal hepatocytes. The FITC Annexin V Apoptosis Detection Kit (Keygen, NJ, China) was used to perform the apoptosis test, which was followed by cell cycle analysis using a flow cytometer.

### 2.11. Recognition of Cell Activity

Isolation and purification of Nf2 were done using an antibody to assess its activity. The Nf2 activity measurements were carried out according to the directions included in the cell activity test kit. To begin an enzymatic reaction, 30 uL of enzyme was introduced to 30 uL of substrate. Standard samples were used to determine the OD value at 450 nm. The relative Nf2 activity in the sample was calculated using the standard curve.

### 2.12. Statistical Analysis

The experimental data were analysed using the statistical programme SPSS 24.0. The results were stated as $\bar{x}\pm s$. Single-factor analysis of variance was employed if the mean of several groups followed a normal distribution, and the LSD technique was used for pairwise comparisons between the groups. Nonparametric tests were employed for data that did not follow a normal distribution, and the Kruskal–Wallis test was used for pairwise comparisons across groups. At a *P* value of <0.05, the differences were considered statistically significant.

## 3. Results

### 3.1. Active Ingredients of SSBE Screening

TCMSP yielded a total of 5 different compounds. Following ADME screening with OB ≥ 30% and DL ≥ 0.18, 20 compounds were identified as SSBE bioactive substances. All five compounds were identified as promising bioactive molecules for future research after HL ≥4 h was optimised. The results of selected 5 compounds from SSBE are presented in Table 1.

### 3.2. DILI's Putative SSBE Targets and the Construction of a Compound-Target Network

185 putative targets linked to 5 compounds of SSBE were collected.

### 3.3. Target Database Establishment of DILI and Common Target Analysis

A total of 707 genes related to DILI were obtained (Figure 1(a)). Through VenNY analysis, 61 common targets of SSBE in the treatment of DILI were obtained (Figure 1(b)).

### 3.4. Common Target Network Analysis and PPI Network of Common Targets

61 common targets were uploaded to the STRING database and the PPI network was generated, with the following conditions: combined score (≥0.4) and species limited to *“Homo sapiens”*. After that, PPI network was established including 59 nodes and 1466 edges by Cytoscape. A larger node and darker color represent the protein that has a greater degree in this network. In addition, a greater combined score of the edge was symbolized by thicker and darker line (Figure 2(a)). We selected 7 targets as critical targets for DILI that have the highest degree score (Figure 2(b)). The key targets that may play a necessary role against DILI include matrix metallopeptidase-9 (MMP9) seed storage protein-1 (SSP1), mitogen-activated protein kinase-14 (MARK14), interleukin-10 (IL-10), interferon-gamma (IFNG), and interleukin-*β* (IL-1*β*).

### 3.5. Enrichment Analysis of GO and KEGG Pathway

Aiming to explore the underlying mechanism of SSBE against DILI, we analysed the enrichment results of the GO term and KEGG pathway executed by DAVID. We divided GO term enrichment results into three parts including biological process (BP), cell compound (CC), and molecular function (MF). The top 10 significant GO terms (BP, MF, and CC) are chosen according to the enrichment score (Figure 3).

After identifying all statistically enriched words, we produced accumulative hypergeometric *P* values and enrichment factors, which we utilised to filter the data. The remaining relevant words were then hierarchically grouped into a tree based on their gene memberships' kappa-statistical similarity. The tree is divided into word clusters using a 0.3 kappa score as a cutoff. The terms within each cluster are exported in the Excel spreadsheet named “Enrichment Analysis.” Cytoscape (v3.1.2) is used to display the network, with a “force-directed” structure with edge bundling for clarity. One phrase from each cluster is chosen as the label for its term description.

Finally, 20 possible signaling pathways are identified, including the IL-17 signaling route, the MAPK, PI3K-Akt, NF-kappa B, and PPAR signaling pathway (Figure 4).

The core targets of the PPI network consisting of MMP9, SSP1, MARK14, IL-10, IFNG, and IL-1*β* found are thought to have a close association with oxidative stress [13–18]. The ingredients of SSBE including asioside, *Sedum sarmentosum* total flavonoids, quercetin, and hyperoside are effective in alleviating liver damage [19]. They mainly alleviate liver injury by regulating oxidative stress, inflammatory signaling pathways, glucose and lipid metabolism disorders, stellate cell activation, and cell regeneration [20]. Nrf2 concerning oxidative or chemical stress of cells is a regulator with a central position [21]. Nrf2-ARE pathway plays a critical role in regulation in a series of biological processes including cellular oxidative stress response, inflammation, tumorigenesis, autophagy, and others. In addition to regulating the expression of II phase detoxifying enzymes and antioxidant enzyme gene, the Nrf2 pathway regulates liver metabolism and detoxification and promotes liver cell regeneration, which is thought to be a critical antioxidant stress pathway [22].

The effect of antioxidant stress is achieved mainly by the nuclear factor erythroid 2-related factor 2 (Nrf2) pathway that plays a central regulating effect in the process of oxidative stress injury concerning cells and the body. In addition, its specific receptor called cytoplasmic protein Kelch-like ECH-associated protein 1 (Keap1) is dissociated first, and then the oxidative stress or electrophilic substances are activated following the stimulation of Keap1. After that, the activated Nrf2 interacts with antioxidant reaction elements (ARE) when it translocates into the nucleus. Moreover, the downstream gene expression was upregulated and thus increased the antioxidant stress ability in cells [23]. We assumed that, in the process of liver injury, SSBE plays an improving role through the Nrf2 signaling pathway by considering the previous research involving SSBE by regulating oxidative stress.

### 3.6. The Anti-Inflammatory Effect of SSBE on the DILI Mouse Model

The distribution of interlobar space of the hepatic lobule was homogeneous and compact in the control group, and there was no edema or inflammatory exudation. The gap between liver cells was dilated in the DILI model group, leukocytes were infiltrated in or around the lobule, and the levels of edema and inflammation were considerably higher than those in the normal group. The SSBE therapy group decreased pancreatic pathological injury to varying degrees. The shift in liver function tests corresponded to the shift in pancreatic pathology. The DILI model group's antioxidation function indexes (GSH, GSH-Px, and SOD) were substantially lower. In terms of the inflammatory response, the DILI model group had substantially higher levels of AST, ALT, and MDA.  Figure 5(a) shows that SSBE decreased inflammatory factors and improved antioxidation function to some extent. The findings revealed that SSBE might prevent the DLLI mice model while also reducing pathological damage and inflammation in the liver (Figure 5(b)).

### 3.7. The Liver Protective Effect of SSBE on the DILI Mouse Model

Flow cytometry analysis showed that, after APAP exposure, SSBE significantly reduced liver cell necrosis (*P* < 0.05) (Figure 6(a)). CCK8 assay showed that SSBE rescued the cell viability of liver cells after exposure to APAP (Figure 6(b)). As shown in Figures 6(c)–6(d), the autophagy of liver cell was inhibited as the concentration of SSBE increased.

### 3.8. The Effect of SSBE on Nrf2 Signaling Pathway on the DLIL Mouse Model

In the animal model experiment, the mRNA level and the expressions of Nrf2 which were proteins in the liver tissue of mice in each group were detected. When compared with the normal group, the mRNA level and the expressions of Nrf2 and ARE proteins in the DILI model group were significantly lower than those in the normal group, and the protein expression and mRNA level improved as the concentration of SSBE increased (Figure 7).

## 4. Discussion

In Chinese herbal formulae, network pharmacology can discover potentially active components, targets, and pharmacological processes of complicated substances [24, 25]. A single SSBE component can interact with many targets, whereas several components can interact with the same target. It is likely that multitarget active compounds have greater clinical efficacy and fewer adverse effects than single-target active chemicals [26, 27].

Traditional Chinese medicine plays a certain role in promoting regeneration and repair of drug-induced liver injury and has unique advantages in DILI treatment. It can play a protective role with multiple components and targets. it has fewer side effects than chemotherapy. SSBE mainly contains flavonoids, cyanosides, alkaloids, triterpenes, sterols, and other compounds, which have anti-inflammatory, liver protection, antirenal fibrosis, antitumor, antioxidant, and other activities. The multicomponent and multitarget network showed the antidrug liver injury effect of SSBE. It shows that there is an interrelation between the constituent targets of SSBE, which is a complex interactive network rather than acting alone. Wang et al. discovered that SSBE had a clear influence on AST, ALT, ALP, GGT/-GT, DBiL, and TBiL levels, as well as increases in ALB and TP levels in serum and ANIT-induced bile flow slowdown for liver damage. The major component of SSBE, *δ*-amyrone, was identified as the efficacious component with hepatoprotective action by boosting Nrf2 antioxidant defense and inhibiting the NF-B inflammatory response [28]. Quercetin has a strong protective effect on the liver among the flavones of SSBE. The antioxidant effect in quercetin mainly showed that it had an obvious protective effect on ischemia-reperfusion injury, and the antioxidant effect in vitro was mainly included. Quercetin can directly eliminate reactive oxygen radicals and play an anti-ischemia-reperfusion injury by upregulation of HO-1 [20]. Hyperin, a main ingredient of SSBE, promotes Nrf2 nuclear translocation by phosphorylating ERK and *P*38, thus activating AREs and upregulating HO-1 to resist oxidative stress injury of human hepatocytes to LO2 caused by H_2_O_2_ [29].

By network pharmacology analysis and experimental validation, this study looked at the pharmacological mechanisms of SSBE in DILI. According to our findings, luteolin, quercetin, isorhamnetin, *ß*-sitosterol, and DFV make up the majority of the chemical makeup of SSBE. Biological activities such as cellular functions, metabolic processes, and oxidative stress responses are among the possible active pathways of SSBE, according to GO word enrichment analysis and KEGG target pathway analysis. Organelles, membranes, and cytoplasm are among the cellular components, as are tiny molecules, cations, and metal ions. It involves a variety of substances such as signal molecules and transcription factors, which is a complex process. And we predicted 7 core targets and the Nrf2 signaling pathway as the main pharmacological mechanisms of SSBE against DILI. The core target of the PPI network is MMP9, SSP1, MARK14, IL-10, IFNG, and IL-1B, which is closely related to oxidative stress [13–18]. Nrf2-ARE pathway is vital in the regulation of cellular oxidative stress response and inflammation.

The Nrf2 signaling pathway is a key endogenous antioxidant stress mechanism, and reactive oxygen species and the oxidative stress response are crucial in the development of liver disorders. Oxidative stress may harm a range of cellular components such as DNA, proteins, and lipids, impacting a variety of organs and systems throughout the body. With numerous targets, the Nrf2 pathway can have a favourable preventive function in the incidence and development of liver disease and postpone the blockage of liver disease progression. Therefore, it is necessary to actively and deeply study the mechanism of the Nrf2 pathway in liver diseases. Our results showed that SSBE was involved in the process of drug-resistant liver injury through the Nrf2 signaling pathway. We also found that SSBE reduced significantly pathological injury and inflammation in the liver. SSBE reduced liver cell necrosis, rescued the cell viability of liver cells, and inhibited the autophagy of liver cells, in which the active compounds of *Sedum sarmentosum* had an effect on improving liver injury. Furthermore, the mRNA level and the expressions of Nrf2 and ARE proteins in liver tissue of mice in the DILI model made by APAP were significantly lower than those in the normal group. As the concentration of SSBE increased, the protein expression and mRNA level increased as the concentration of SSBE improved (Figure 7(a)). We can conclude that the Nrf2-ARE pathway is vital in the effect of improving liver injury by SSBE.

Furthermore, KEGG target pathways reveal that possible signaling pathways such as the IL-17 signaling route, MAPK signaling pathway, PI3K-Akt signaling pathway, NF-kappa B signaling network, and PPAR signaling pathway are linked to the creation and progression of liver damage. The key targets of SSBE antiliver injury active components are distributed in different pathways, which can coordinate each pathway to play an antiliver injury role. These pathways can all serve as directions for further research in the future.

There were some flaws in this study, as well as certain areas that need more research. These include the need for a more thorough investigation of protein interactions and predicted monomers, as well as an increase in the DILI chip's sample size from the database. Despite this, the possibility of investigating DILI therapy with traditional SSBE prescription based on network pharmacology was verified in this investigation. This reduces the amount of time and money spent on exploration as well as the expense of scientific study. This research suggests that more research on monomers and associated transcription factors with potential therapeutic effects on DILI might be done in the future. This might pave the way for a breakthrough in the treatment of DILI with traditional Chinese medicine.

## 5. Conclusion

In summary, the network pharmacology and in vivo experimental results in this study indicated that SSBE reduced the inflammatory response caused by APAP in a DLII model and protected liver tissue. 61 potentially active components of SSBE in DILI treatment were discovered using network pharmacology techniques and drug toxicity risk assessment. Furthermore, the Nrf2 signaling pathway was found to play an important regulatory role in the mechanism of DILI in the treatment of SSBE.

## Figures and Tables

**Figure 1:** Venn diagram of DILI gene and target of drug and disease intersection.

**Figure 2:** Protein-protein interaction network and the key subnetwork.

**Figure 3:** The key subnetwork of PPI.

**Figure 4:** The KEGG pathway enrichment analysis of common targets.

**Figure 5:** Liver tissue-related detection. (a) HE section of the liver tissue in different groups; (b) the contents of GSH, GSH-PX, AST, ALT, SOD, and MDA in the liver tissue in different groups. ^*∗∗*^*P* < 0.05 versus the normal group.

**Figure 6:** The liver protective effect of SSBE on the DILI mouse model. (a) Flowchart of apoptosis/necrosis in different groups; (b) cell viability in different groups by CCK8 assay; (c) expression of cell proteins in different groups, including LC3I and LC3II; (d) fold sham in different groups. ^*∗∗*^*P* < 0.05 versus the normal group.

**Figure 7:** The effect of SSBE on the Nrf2 signal pathway in the DILI mouse model. (a), (b) Expression of Nrf2, ARE, and NADPH in different groups. (c) Expression of Nrf2 and ARE. (d, e) Corresponding fold sham of Nrf2 and ARE. ^*∗∗*^*P* < 0.05 versus the normal group.

**Table 1:** A list of the final selected active compounds of SSBE.

Molecule ID	Molecule name	OB (%)	DL	HL
MOL001792	DFV	32.76	0.18	17.89
MOL000354	Isorhamnetin	49.60	0.31	14.34
MOL000358	Beta-sitosterol	36.91	0.75	5.36
MOL000006	Luteolin	36.16	0.25	15.94
MOL000098	Quercetin	46.43	0.28	14.40

## Data Availability

The data used to support the findings of this study are available from the corresponding author upon request.

## References

[1] Kuna L., Bozic I., Kizivat T. (2018). Models of drug induced liver injury (DILI) - current issues and future perspectives. *Current Drug Metabolism*.

[2] Kullak-Ublick G. A., Andrade R. J., Merz M. (2017). Drug-induced liver injury: recent advances in diagnosis and risk assessment. *Gut*.

[3] Wan D., Chen Y., Wang J. (2010). Determination of total flavonoids in three Sedum crude drugs by UV-Vis spectrophotometry. *Pharmacognosy Magazine*.

[4] Huang L., Cheng Y., Huang K., Zhou Y., Ma Y., Zhang M. (2018). Ameliorative effect of Sedum sarmentosum bunge extract on tilapia fatty liver via the PPAR and P53 signaling pathway. *Scientific Reports*.

[5] Lu H., Cheng S., Wu C. (2019). Sedum sarmentosum bunge extract alleviates inflammation and kidney injury via inhibition of M1-macrophage polarization. *Phytomedicine*.

[6] Hopkins A. L. (2008). Network pharmacology: the next paradigm in drug discovery. *Nature Chemical Biology*.

[7] Cai F.-F., Zhou W.-J., Wu R., Su S.-B. (2018). Systems biology approaches in the study of Chinese herbal formulae. *Chinese Medicine*.

[8] Li S., Zhang B., Zhang N. (2011). Network target for screening synergistic drug combinations with application to traditional Chinese medicine. *BMC Systems Biology*.

[9] Ru J., Li P., Wang J. (2014). TCMSP: a database of systems pharmacology for drug discovery from herbal medicines. *Journal of Cheminformatics*.

[10] Ru J., Li P., Wang J. (2014). TCMSP: a database of systems pharmacology for drug discovery from herbal medicines. *Journal of Cheminformatics*.

[11] Yu G., Luo Z., Zhou Y. (2019). Uncovering the pharmacological mechanism of Carthamus tinctorius L. on cardiovascular disease by a systems pharmacology approach. *Biomedicine & Pharmacotherapy*.

[12] Wang W., Liu T., Yang L. (2019). Study on the multi-targets mechanism of triphala on cardio-cerebral vascular diseases based on network pharmacology. *Biomedicine & Pharmacotherapy*.

[13] Dwir D., Giangreco B., Xin L. (2019). MMP9/RAGE pathway overactivation mediates redox dysregulation and neuroinflammation, leading to inhibitory/excitatory imbalance: a reverse translation study in schizophrenia patients. *Molecular Psychiatry*.

[14] Quong J., Eppenberger-Castori S., Moore D. (2002). Age-dependent changes in breast cancer hormone receptors and oxidant stress markers. *Breast Cancer Research and Treatment*.

[15] Weber D., Stuetz W., Buerkle A., Grune T. (2017). Oxidative stress biomarkers in the MARK-AGE Study. *Free Radical Biology and Medicine*.

[16] Deepali S., Kumar V., Chetna S. (2017). IFN-*γ* regulates xanthine oxidase-mediated iNOS-independent oxidative stress in maneb- and paraquat-treated rat polymorphonuclear leukocytes. *Molecular and Cellular Biochemistry*.

[17] Tanaka Y., Hiroshi U., Akiko H., Masutaka F. (2018). Tryptophan photoproduct FICZ upregulates IL1A, IL1B, and IL6 expression via oxidative stress in keratinocytes. *Oxidative Medicine & Cellular Longevity*.

[18] Kaur K., Sharma A., Dhingra S., Singal P. (2006). Interplay of TNF-*α* and IL-10 in regulating oxidative stress in isolated adult cardiac myocytes. *Journal of Molecular and Cellular Cardiology*.

[19] Lian L.-H., Jin X., Wu Y.-L., Cai X. F., Lee J. J., Nan J.-X. (2010). Hepatoprotective effects of Sedum sarmentosum on D-galactosamine/lipopolysaccharide-induced murine fulminant hepatic failure. *Journal of Pharmacological Sciences*.

[20] Atef Y., El-Fayoumi H. M., Abdel-Mottaleb Y., Mahmoud M. F. (2017). Quercetin and tin protoporphyrin attenuate hepatic ischemia reperfusion injury: role of HO-1. *Naunyn-Schmiedeberg’s Archives of Pharmacology*.

[21] Tonelli C., Chio I. I. C., Tuveson D. A. (2018). Transcriptional regulation by Nrf2. *Antioxidants and Redox Signaling*.

[22] Buendia I., Michalska P., Navarro E., Gameiro I., Egea J., León R. (2016). Nrf2-ARE pathway: an emerging target against oxidative stress and neuroinflammation in neurodegenerative diseases. *Pharmacology & Therapeutics*.

[23] Ahmed S. M. U., Luo L., Namani A., Wang X. J., Tang X. (2017). Nrf2 signaling pathway: pivotal roles in inflammation. *Biochimica et Biophysica Acta - Molecular Basis of Disease*.

[24] Wang X., Shen Y., Wang S. (2017). PharmMapper 2017 update: a web server for potential drug target identification with a comprehensive target pharmacophore database. *Nucleic Acids Research*.

[25] Zhao Y.-l., Wei S., Niu M. (2016). A network pharmacology approach to discover active compounds and action mechanisms of San-Cao Granule for treatment of liver fibrosis. *Drug Design, Development and Therapy*.

[26] Mao Y., Hao J., Jin Z.-Q. (2017). Network pharmacology-based and clinically relevant prediction of the active ingredients and potential targets of Chinese herbs in metastatic breast cancer patients. *Oncotarget*.

[27] Wu R., Li X.-Y., Wang W.-H. (2019). Network pharmacology-based study on the mechanism of bushen-jianpi decoction in liver cancer treatment. *Evidence-based Complementary and Alternative Medicine*.

[28] Wang G.-W., Zhang X.-L., Wu Q.-H. (2019). The hepatoprotective effects of Sedum sarmentosum extract and its isolated major constituent through Nrf2 activation and NF-*κ*B inhibition. *Phytomedicine*.

[29] Xing H.-Y., Liu Y., Chen J.-H., Sun F.-J., Shi H.-Q., Xia P.-Y. (2011). Hyperoside attenuates hydrogen peroxide-induced L02 cell damage via MAPK-dependent Keap1-Nrf2-ARE signaling pathway. *Biochemical and Biophysical Research Communications*.

